RETRACTED

# Ablation of Basic Leucine Zipper Transcription Factor ATF-Like Potentiates Estradiol to Induce Atopic Dermatitis

**DOI:** 10.1155/2022/7024669

**Published:** 2022-09-16

**Authors:** Peng Zhang, Luhao Liu, Xingqiang Lai, Rongxin Chen, Yuhe Guo, JunjieMa, Wenhao Chen, Zheng Chen

**Affiliations:** ^1^Organ Transplant Center, The Second Affiliated Hospital of Guangzhou Medical University, Guangzhou, 511447 Guangdong, China; ^2^Immunobiology & Transplant Science Center, Houston Methodist Research Institute, Texas Medical Center, Houston, TX 77030, USA

## Abstract

**Background:**

Atopic dermatitis (AD) is an inflammatory and immune skin disorder. Basic leucine zipper transcription factor ATF-like (BATF) plays a key role in regulating the differentiation and functions of lymphocytes. However, the mechanism underlying the transcriptional regulation of BATF on AD is still not well understood.

**Methods:**

BATF knockout (BATF^–/–^) and C57BL/6(B6) mice were used for the development of spontaneous dermatitis. 17*β*-Estradiol was injected intraperitoneally to induce AD. The lesioned tail skin of the mice was stained with hematoxylin and eosin to analyze the pathological characteristics. Impaired skin barrier function was assessed by measuring the transepidermal water loss (TEWL). The skin epithelial barrier indicators and cytokine mRNA levels were quantified by real-time quantitative PCR. The total serum immunoglobulin E (IgE) levels were measured by enzyme-linked immunosorbent assay (ELISA). T lymphocytes were analyzed using flow cytometry.

**Results:**

Ablation of BATF led to the spontaneous development of AD only in female mice and not in male mice. BATF deletion led to elevated serum levels of IgE and increased infiltration of eosinophils, neutrophils, and lymphocytes and promoted cytokine production including IL-4, IL-22, IL-1*β*, IFN-*γ*, and TNF-*α* in the lesioned tail skin of the mice. The mRNA expression levels of filaggrin and loricrin significantly decreased, while S100A8 and S100A9 increased in female BATF^–/–^ mice. BATF-deficient female mice were found to increase proliferation and IL-5 production by skin-infiltrating CD4^+^ T cells which implies Th2 activation. Moreover, AD was successfully induced only in the estradiol-treated BATF-deficient male mice and not in WT male mice. Estradiol enhanced the allergic and immunological responses to dermatitis primarily by triggering Th2-type immune responses via enhanced serum IgE and inflammatory cytokine levels in the male BATF^–/–^ mice.

**Conclusion:**

The study concluded that BATF potentiates estradiol to induce mouse atopic dermatitis via potentiating inflammatory cytokine releases and Th2-type immune responses and may have important clinical implications for patients with AD.

RETRACTED

## 1. Introduction

Atopic dermatitis (AD) is a chronic relapsing and remitting inflammatory skin disease affecting one in 10 people in their lifetime. AD is caused by a complex interaction of multiple factors such as immune dysregulation, epidermal gene mutations, and environmental factors. Approximately 80% of AD cases have allergic reactions and are categorized as extrinsic or allergic AD (1). Such patients are characterized by elevated levels of total serum immunoglobulin E (IgE) and the presence of specific IgE for environmental and food allergens. AD without the presence of an allergen is called intrinsic AD. AD is known to be primarily a T cell-driven disease, with a dominant T helper (Th) type 2 immune response with increased levels of IL-4, IL-13, and IL-31 and additional activation of Th22,Th17/I L-23, and Th1 cytokine pathways (2–4).

Basic leucine zipper transcription factor ATF-like (BATF) belongs to the activator protein 1 family of transcription factors and is highly expressed in lymphocytes (5). BATF plays a key role in regulating the differentiation and functions of T cells, B cells, and dendritic cells. In Th cells, BATF is required for Th9, Th17, and T follicular helper (Tfh) cell differentiation (6–9). BATF deficiency in T cells can lead to impaired T cell-mediated immune response function, resulting in dermatitis, allergic asthma, and autoimmunity (10–14). Early-onset AD is characterized by Th2/Th17/Th22-centered inflammation (15). BATF is required for the differentiation of IL-17-producing T helper (Th17) cells, which comprise a distinct subset of CD4^+^ T cells that produce inflammatory responses in host defense against the development of autoimmune diseases (16, 17). Moreover, BATF was reported to be a potential biomarker for distinguishing allergic and irritant contact dermatitis affecting human skin (18). However, the underlying mechanism by which BATF affects AD is still unclear.

In the present study, the role of BATF in AD development was examined. The study indicated that BATF deletion led to spontaneous development of AD only in female mice and not in male mice. BATF deletion was associated with elevated serum IgE levels, enhanced cytokine production in skin tissues, and increased proliferation and IL-5 production by skin-infiltrating CD4^+^ T cells. Furthermore, male wild-type (WT) and BATF-deficient mice were treated with estradiol or sesame oil (vehicle control) for 20 weeks. It was found that AD was successfully induced in the estradiol-treated BATF-deficient mice, but not in the estradiol-treated WT and sesame oil-treated BATF-deficient mice. Therefore, it can be concluded that the deletion of BATF stimulates estradiol to induce AD. The findings from this study elucidate the AD development at the transcriptional level.

RETRACTED

## 2. Methods

### 2.1. Animals

C57BL/6(B6) and BATF^–/–^ mice were supplied by the Jackson Laboratory (Bar Harbor, ME, USA). BATF^–/–^ mice were generated by the homologous recombination, deleting exons 1 and 2 of the *Batf* gene on the pure 129SvEv genetic background, as described in a previous study (16). Female mice were used to observe the development of spontaneous dermatitis without any treatment. Male mice were subjected to hormonal treatment for induction of dermatitis. The mice were housed in a limited-access rodent facility with up to five mice per polycarbonate cage. The mice were bred and maintained in a specific pathogen-free facility at Houston Methodist Research Institute in Houston, Texas, under a 12 h light/12 h dark cycle (08:00–20:00 h light and 20:00–08:00 h dark) at 23 ± 2°C and 50 ± 10% humidity with free access to food and water. All the animal experiments in this study were approved by the Houston Methodist Animal Care Committee following the guidelines of the institutional committee for animal care and use.

### 2.2. Reagents

Flow cytometry was performed using the following fluorochrome-conjugated antibodies: CD3e Monoclonal Antibody (145-2C11) (Thermo Fisher Scientific, Waltham, USA), PE/Cyanine7 anti-mouse CD4 Antibody (BioLegend, San Diego, USA), anti-mouse CD8a Antibody (BioLegend, San Diego, USA), CD25 Monoclonal Antibody (PC61.5) (Thermo Fisher Scientific, Waltham, USA), PE/Cyanine7 anti-mouse TCR *β* chain Antibody (BioLegend, San Diego, USA), Purified anti-mouse/human IL-5 Antibody (BioLegend, San Diego, USA), Ki-67 Monoclonal Antibody (SolA15)(Thermo Fisher Scientific, Waltham, USA), and FOXP3 Monoclonal Antibody (FJK-16s) (Thermo Fisher Scientific, Waltham, USA). A Foxp3 Transcription Factor Staining Set was purchased from eBioscience (Thermo Fisher Scientific, Inc.). A Zombie Aqua Fixable Viability Kit was obtained from BioLegend. Collagenase-IV, 17*β*-estradiol (E2), DNase I, sesame oil, phorbol 12-myristate 13-acetate (PMA), and ionomycin were purchased from Sigma-Aldrich (St. Louis, MO, USA).

### 2.3. Estradiol Treatment

WT B6 and BATF^–/–^ male mice were injected intraperitoneally with either 1 mg/kg 17*β*-estradiol or sesame oil (vehicle control) every 3 days to determine the effect of estradiol on AD in BATF^–/–^ mice. The estradiol treatment was started when the mice were 4 weeks old and stopped when they were 24 weeks old.

### 2.4. Scoring of the Severity of Skin Inflammation

The clinical severity of skin inflammation on the tail of the mice was scored according to the macroscopic diagnostic criteria as previously described (19). Briefly, the severity of dermatitis was assessed according to four symptoms: (i) erythema/hemorrhage, (ii) scarring/dryness, (iii) edema, and (iv) excoriation/erosion. Each symptom was scored on a scale of 0 to 3 (none, 0; mild, 1; moderate, 2; and severe, 3). The total score for each mouse was calculated as the sum of the individual scores for each parameter and ranged from 0 to 12.

RETRACTED

### 2.5. Measurement of Transepidermal Water Loss (TEWL)

Transepidermal water loss (TEWL) in 28-week-old mice was measured with a Tewameter® TM210 (EnviroDerm, Evesham, UK) under sevoflurane anesthesia, as previously described (20). Briefly, TEWL measurements were conducted by placing a probe against the surface of the tail skin over a 1 min period. TEWL was recorded at an ambient temperature of 20–26°C and a humidity of 45–55%. The average of three readings per mouse was calculated, and measurements were recorded as grams per meter square per hour (g/m^2^/h).

### 2.6. Histological Analysis

The tail skins of the mice were sectioned and stained with hematoxylin and eosin. Briefly, mice from each group were deeply anesthetized with sodium pentobarbital (50 mg/kg IP), and their tail skin tissues were quickly sectioned. Tail skin biopsies were fixed overnight in fresh 4% PFA at 4°C, then washed in TBS, embedded in paraffin, and cut into 5 *μ*m sections using a rotatory microtome (Finesse 325; Thermo Shandon Co., UK). The cut sections were deparaffinized and stained with hematoxylin (Merck, Darmstadt, Germany) and 1% eosin (Sigma-Aldrich Co.). The histological images were examined using a microscope equipped with a digital camera (BX51; Olympus Co., Tokyo, Japan) and DP2-BSW analysis software (Olympus Co). The infiltration of individual inflammatory cells into the skin was quantified using a scoring system as previously described (21). The total number of cells was quantified by counting the number of cells in 1,000 high-power fields (HPF) of view, and the average number of cells was calculated across 20 HPFs (22). Epidermal thickness was measured on at least 15 different random fields per specimen.

### 2.7. Quantitation of Serum Total IgE

Total IgE levels in the serum of 28-week-old BATF^–/–^ mice and WT mice were measured by enzyme-linked immunosorbent assay (ELISA). Briefly, plates were coated with 2 *μ*g/mL IgE (BioLegend, San Diego, CA, USA) at 4°C overnight. The plates were blocked with 1% BSA in PBS for 1 h the following day and then coated with samples of serum from the mice. Further, IgE-biotin conjugate (2.0 *μ*g/mL) and streptavidin-HRP (1: 1,000; BioLegend) were sequentially added, and the reaction was catalyzed using tetramethylbenzidine as a substrate (BioLegend). Serum total IgE concentration was determined from a standard curve generated using a known concentration of mouse IgE supplied by the manufacturer.

RETRACTED

### 2.8. Quantitative Real-Time Polymerase Chain Reaction

Total RNA was extracted from whole tail skin using an Ambion RNA Isolation Kit (Thermo Fisher Scientific, Waltham, MA, USA). The RNA quantity was measured using a NanoDrop ND-2000 spectrophotometer (Thermo Fisher Scientific). The PrimeScript™ 1st Strand cDNA Synthesis Kit (Roche Diagnostics GmbH, Mannheim, Germany) was used to synthesize cDNA according to the protocol provided by the manufacturer. A real-time quantitative polymerase chain reaction (qPCR) was performed using SYBR Green Master Mix (TAKARA, Tokyo, Japan).  Table 1 provides a list of the specific primers for each target gene. The 2 (-delta C (T)) method was used to analyze the relative changes in expression of target genes as per the protocol given by the manufacturer (CFX96 Touch Real-Time PCR Detection System; Bio-Rad). The primers were denatured at 95°C for 5 min before PCR amplification and then subjected to the following amplification program: 95°C for 10 s, 60°C for 20 s, and 72°C for 20 s for each cycle for a total of 44 cycles, followed by a final elongation at 72°C for 5 min. The gene expression was expressed in arbitrary units relative to the expression of GAPDH.

### 2.9. Isolation of Infiltrating Mononuclear Cells from Tail Skins

Whole tail skin was minced and digested in Dulbecco's Modified Eagle Medium (DMEM, Gibco) containing 5% FBS, 2.5 mg/mL collagenase-IV, and 1 mg/mL DNase I, at 37°C for 1 h. The digested tissue was then filtered through a 70 *μ*m cell strainer, followed by Percoll gradient centrifugation (37% and 70%). The mononuclear cells in the interphase were collected, washed, and resuspended in a DMEM culture medium.

### 2.10. Flow Cytometry Analysis

Splenocytes and infiltrating mononuclear cells from tail skins were preincubated using Zombie Aqua Viability Kit for 10 min and subsequently stained with fluorochrome-labeledanti-CD3, anti-CD4, anti-CD8, anti-CD25, anti-TCR-*β*, anti-ki-67, and anti-Foxp3 antibodies for 30 min at 4°C. The Foxp3 Transcription Factor Staining Set (Thermo Fisher Scientific) was used for Foxp3 intracellular staining. The cells were stimulated with phorbol 12-myristate 13-acetate (PMA, 50 ng/mL) and ionomycin (550 ng/mL) in the presence of GolgiStop (BD Biosciences) for 4 h to measure IL-5 expression levels. Further, the cells were fixed and permeabilized with Cytofix/Cytoperm solution (BD Biosciences) and then stained with fluorochrome-conjugated anti-IL-5. The stained cells were analyzed in the LSR II flow cytometer (Becton Dickinson), and the resulting data were processed using FlowJo v10 software (Tree Star, Inc.).

RETRACTED

### 2.11. Statistical Analysis

The data were expressed as mean ± standard error and analyzed by unpaired Student's *t*-tests, one-way analysis of variance (ANOVA), or two-way ANOVA with a Bonferroni post hoc test using Prism version 6.0 software (GraphPad Software Inc., San Diego, CA, USA). All *P* values less than 0.05 were considered statistically significant. *P* values are denoted in figures as follows: n.s., *P* > 0.05; ∗, *P* < 0.05; ∗∗, *P* < 0.01; and ∗∗∗, *P* < 0.001.

## 3. Results

### 3.1. Development of Atopic Dermatitis in Female BATF-Deficient Mice

The transcriptional control of the inflammatory responses to AD has not been well elucidated. In the present study, when compared with female WT B6 mice under specific-pathogen-free conditions, all the female BATF^–/–^ mice spontaneously developed ichthyosis-like dermatitis with distinct symptoms such as edema, hyperlinearity, erosions, crusts, scales, and lichenification on their tail skin before 16 weeks of age (Figure 1(a)). In addition to dermatitis, skin lesions were also observed on the ears, faces, and necks of most of the female BATF^–/–^ mice (Figure 1(b)). The longitudinal scoring of the severity of skin inflammation indicated the development of AD in female BATF^–/–^ mice (Figure 1(c)). In 8-week-old female BATF^–/–^ mice, early ichthyosis-like skin lesions were initially observed on the tail skin. By 16 weeks, a majority of female BATF^–/–^ mice had developed varying degrees of dermatitis, which progressed to severe dermatitis by 28 weeks. However, the male BATF^–/–^ mice did not develop dermatitis (data not shown). When compared with the tail skins from age-matched female WT B6 mice, the histology of tail skins from the female BATF^–/–^ mice at 28 weeks of age revealed a thickening of the epidermis with acanthosis, hypogranulosis, and mild hyperkeratosis (Figure 1(d)). Skin thickening is the first indication of skin irritation and local inflammation. The epidermal thickness of the tail skins of female BATF^–/–^ mice showed a fourfold increase at 28 weeks of age when compared with that of the tail skins of the female WT B6 mice (Figure 1(e)).

An impaired skin barrier is one of the basic features of AD and can be assessed by measuring TEWL (23, 24). The TEWL values in the tail skins of 28-week-old female BATF^–/–^ mice significantly increased when compared with those in the tail skins of female WT B6 mice, indicating skin barrier dysregulation in the female BATF^–/–^ mice (Figure 1(f)). Altogether, female BATF^–/–^ mice spontaneously developed ichthyosis-like dermatitis in an age-dependent manner.

RETRACTED

### 3.2. Increase in the Serum IgE Levels and Cytokine Production in Skin Tissues of Female BATF^–/–^ Mice with AD

For a better understanding of the immunological mechanisms of AD in this study, female BATF^–/–^ and WT B6 mice were euthanized at 28 weeks of age for *ex vivo* analysis. The spleen and regional draining lymph nodes to the skin lesions, including branchial, axillary, and inguinal lymph nodes, were found to be significantly enlarged in the female BATF^–/–^ mice when compared with those in the female WT B6 mice (Figure 2(a)). Moreover, ELISA tests highlighted that at 28 weeks, the total serum IgE levels, which are an essential marker of AD (25), in female BATF^–/–^ mice with dermatitis were significantly elevated when compared with those in WT controls (Figure 2(b)). These findings indicated an enhanced allergic response in female BATF^–/–^ mice with dermatitis.

Histopathologic analysis of the lesioned tail skin at 24 weeks revealed profound infiltration by eosinophils (*P* < 0.01), neutrophils (*P* < 0.05), and lymphocytes (*P* < 0.01) into the dermis (Figure 2(c)). Further, the gene expression levels of skin barrier proteins and cytokines in skin tissues were analyzed. Filaggrin and loricrin are key components for maintaining normal skin epithelial barrier function (26). The mRNA expression levels of filaggrin and loricrin in the tail skins of female BATF^–/–^ mice significantly decreased when compared with those in the tail skins of the WT controls. The expression levels of mRNAs encoding calcium-binding proteins, namely, S100A8 and S100A9, were also measured. These proteins act as neutrophil chemotaxis and strong adhesion inducers during inflammatory responses. The data from this study revealed elevated mRNA expression levels of S100A8 and S100A9 in the lesioned tail skin of the female BATF^–/–^ mice when compared with those in the tail skin of the WT controls (Figure 2(d)).

Further, the expression levels of cytokine mRNAs, including IL-4, IL-5, IL-22, IL-1*β*, IFN-*γ*, and TNF-*α*, rapidly increased in the tail skins of female BATF^–/–^ mice when compared with those in the tail skins of the WT controls (Figure 2(e)). Altogether, the study results indicated that AD in female BATF-deficient mice was associated with increased serum IgE levels and cytokine production in skin tissues.

### 3.3. Increased Proliferation and IL-5 Production by Skin-Infiltrating CD4^+^ T Cells in the Female BATF^–/–^ Mice with AD

For a better understanding of the immunological mechanisms of AD in this study, tail skin-infiltrating mononuclear cells were isolated from 28-week-old female BATF^–/–^ and WT mice for flow cytometric analysis. Splenocytes were also harvested and analyzed. There was no significant difference in the frequencies of CD4^+^ and CD8^+^ T cells among CD3^+^ splenocytes, nor in the frequency of Foxp3^+^ cells within the CD4^+^ subset of splenocytes, between the female BATF^–/–^ and WT mice (Figures 3(a) and 3(b)). The frequencies of Ki67^+^ and IL-5^+^ cells in the CD4^+^splenocytes of female BATF^–/–^ mice were statistically higher than those in the CD4^+^ splenocytes of female WT mice (Figures 3(c) and 3(d)).

RETRACTED

The differences in the phenotype and frequency of tail skin-infiltrating CD4^+^ T cells were evident between the female BATF^–/–^ mice and female WT mice. In the female BATF^–/–^ mice, CD4^+^ T cells accounted for more than 80% of the skin-infiltrating T cells, whereas in WT female mice, approximately 50% of skin-infiltrating T cells were CD4^+^ T cells (Figure 3(a)). The skin-infiltrating CD4^+^ T cells in the female BATF^–/–^ mice had decreased levels of regulatory T (Treg) cell marker Foxp3 expression and increased levels of proliferative marker Ki67 expression when compared with those in the female WT mice (Figures 3(b) and 3(c)). The salient feature of the BATF^–/–^ female mice was that more than 13% of skin-infiltrating CD4^+^ T cells produced IL-5. On the contrary, less than 2% of skin-infiltrating CD4^+^ T cells produced IL-5 in the female WT mice (Figure 3(d)). Thus, AD in female BATF^–/–^ mice was associated with increased proliferation and IL-5 production by skin-infiltrating CD4^+^ T cells.

### 3.4. Estradiol Induced AD in BATF^–/–^ Male Mice

Spontaneous AD was developed only in the female BATF^–/–^ mice and not in the male BATF^–/–^ mice. In this study, the role of estrogen in inducing AD in BATF-deficient mice was investigated. The male WT B6 and BATF^–/–^ mice were injected intraperitoneally with either 1 mg/kg 17*β*-estradiol or sesame oil (vehicle control) every 3 days. The estradiol treatment was started when the mice were 4 weeks old and stopped when they reached 24 weeks of age. As shown in Figure 4(a), estradiol treatment induced AD, especially in the tail skins of male BATF^–/–^ mice. However, none of the estradiol-treated WT or sesame oil-treated male BATF^–/–^ mice developed AD. Moreover, longitudinal scoring of the severity of skin inflammation indicated that estradiol induced AD in the male BATF^–/–^ mice in a time-dependent manner (Figure 4(b)). The histology of tail skins from the estradiol-treated male BATF^–/–^ mice at 24 weeks of age highlighted the thickening of the epidermis, with acanthosis, hypogranulosis, mild hyperkeratosis, and more inflammatory cell infiltration when compared with the tail skins from the estradiol-treated WT controls and sesame oil-treated male BATF^–/–^ mice (Figure 4(c)). ELISA revealed that the total serum IgE levels of the estradiol-treated male BATF^–/–^ mice significantly increased, indicating that estradiol led to enhanced allergic and immunological responses to dermatitis in the male BATF^–/–^ mice (Figure 4(d)).

RETRACTED

Finally, the variations in the levels of inflammatory cytokines in the tail skin of the mice were examined. A significant increase in mRNA levels of IL-4, IL-5, IL-1*β*, and IFN-*γ* was observed in the estradiol-treated male BATF^–/–^ mice; however, no substantial differences were observed in the other two groups. Estradiol mainly led to an increase in Th2 cytokines in the male BATF^–/–^ mice (Figure 4(e)). These findings indicated that estradiol induced AD and increased serum IgE levels and cytokine production in male BATF^–/–^ mice.

## 4. Discussion

AD is a chronic inflammatory skin disease characterized by pruritus, barrier disruption, and inflammation including type 2 cytokine production induced mainly by immune dysregulation. The transcriptional programs regulating the development of AD have not been well studied. In the present study, it was demonstrated that AD spontaneously developed only in female BATF-deficient mice and not in the male BATF-deficient mice. Further, a mechanistic analysis revealed that the female BATF*-*deficient mice with AD exhibited elevated levels of serum IgE, enhanced cytokine production in skin tissues, and increased proliferation and IL-5 production by skin-infiltrating CD4^+^ T cells. Therefore, AD in BATF-deficient female mice led to allergic reactions, and IL-5-producing Th cells may be responsible for the development of skin lesions. Another major finding of this study was that the male BATF-deficient mice treated with estradiol developed AD; however, their WT counterparts did not develop AD. Therefore, it can be stated that BATF deletion stimulates estradiol to induce AD.

BATF is a key transcriptional factor controlling the differentiation of Th9, Th17, and Tfh cells (27–29). Therefore, the absence of BATF results in impaired T cell-mediated responses, leading to autoimmunity, allergic asthma, and chronic infection. Thus, BATF plays a crucial role in regulating Th2-type immune responses, depending on the presence of its binding sites on Th2 cells (30). For instance, recently, Kuwahara *et al.* (31) showed that the BATF-IRF4 complex promotes the production of Th2 cytokines, whereas the Bach2-BATF complex antagonizes the recruitment of the BATF-IRF4 complex to AP-1 motifs and suppresses the production of Th2 cytokines. In this study, it was demonstrated that AD in the female BATF*-*deficient mice led to allergic reactions, indicating the involvement of the Th2 pathway. It was evident that the expressions of genes encoding Th2 cytokines IL-4 and IL-5 significantly increased in tail skins of the female BATF-deficient mice with AD, although the expression of the gene encoding Th1 cytokine IFN-*γ* also increased. Skin-infiltrating T cells in these mice were primarily CD4^+^ and produced a significant amount of IL-5. The study findings demonstrated that BATF is a repressor of Th2 response, and the female mice developed Th2 cell-mediated allergic AD in the absence of BATF.

RETRACTED

In human subjects, AD, especially intrinsic AD, is predominant in females (32). In this study, allergic AD was spontaneously developed only in the female BATF-deficient mice and not in the male BATF-deficient mice. Therefore, the role of estrogen in inducing AD was investigated in the present study. It was found that estradiol treatment successfully induced AD in male BATF-deficient mice, but not in WT male mice. These findings indicate that allergic AD in BATF-deficient mice is associated with estrogen. Further studies are required to assess the sex-specific association between inflammatory reaction and AD development.

In conclusion, the role of BATF in AD development was elucidated. BATF restricted the production of cytokines, including IL-4, IL-22, IL-1*β*, IFN-*γ*, and TNF-*α* in the tail skin of the female mice. The deletion of BATF led to a rapid increase in all the cytokines mentioned above. BATF deletion was also associated with elevated serum IgE levels and infiltration of eosinophils, neutrophils, and lymphocytes. Moreover, skin-infiltrating CD4^+^ T cells in BATF^–/–^ female mice overexpressed IL-5 which implies Th2 activation. IL-5 was shown to be a potential therapeutic target for the treatment of AD (33). The results in the present study indicated the inhibition of Th2-type immune response in AD by BATF. This highlights the role of BATF in regulating the Th response to inflammatory skin disorders. On the contrary, AD was successfully induced in the estradiol-treated BATF-deficient male mice. Estradiol enhanced the allergic and immunological responses to dermatitis mainly by increased activation of Th2 cells that enhanced serum IgE and inflammatory cytokine levels in the male BATF^–/–^ mice.

Overall, this study provides novel insights into the mechanisms underlying potentiation of estradiol by BATF to induce mouse atopic dermatitis by triggering Th2-type immune responses via enhancing the release of inflammatory cytokines. These results may have important clinical implications for patients with AD.

RETRACTED

## Figures and Tables

**Figure 1:** BATF-deficient female mice develop spontaneous atopic dermatitis. (a) A representative image of tails from 3 female BATF^–/–^ (*Batf*^–/–^F) mice at 24–28 weeks of age and from one 26-week-old female WT (WT F) mouse. (b) Representative images of the facial and cervical skins from 24–28-week-old female BATF^–/–^ and WT mice. (c) Macroscopic scores of dermatitis in female BATF^–/–^ (*n* = 24) and WT (*n* = 22) mice at the indicated ages. Statistical significance was determined by two-way analysis of variance. (d) Representative H&E-stained tail skin sections from 28-week-old female BATF^–/–^ and WT mice. Scale bars: 200 *μ*m (400× magnification) and 100 *μ*m (200× magnification). (e) Epidermal thickness of the mouse tail skins was assessed by morphometric analysis. Data are shown as mean ± standard error of the mean (SEM) of the epidermal thickness of the tail skins, with 10 mice per indicated group at 28 weeks of age.(f) Transepidermal water loss (TEWL) of the tail skins, with 22 mice per indicated group at 28 weeks of age. ^∗^*P* < 0.05, ^∗∗^*P* < 0.01, and ^∗∗∗^*P* < 0.001, compared with the WT group.

**Figure 2:** Serum IgE levels and cytokine production in skin tissues are increased in female BATF^–/–^ mice. (a) A representative image of spleens and indicated lymph nodes from 20-week-old BATF^–/–^ and WT female mice. (b) Total serum IgE levels detected by enzyme-linked immunosorbent assay (ELISA) from 28-week-old female BATF^–/–^ and WT mice (*n* = 20 per group). (c) Dermal eosinophil, neutrophil, and lymphocyte counts per high-power field (HPF) in lesioned tail skins of 28-week-old female BATF^–/–^ and WT mice (*n* = 6 per group). (d) Decreased mRNA expression of filaggrin and loricrin combined with increased mRNA expression of S100 family proteins in the tail skin. (e) Relative mRNA expressions of IL-4, IL-5, IL-22, IL-1*β*, IFN-*γ*, and TNF-*α* in tail skins from 28-week-old female BATF^–/–^ and WT mice (*n* = 5 per group). Data are shown as mean ± standard deviation (SD) and are representative of three independent experiments. ^∗^*P* < 0.05, ^∗∗^*P* < 0.01, and ^∗∗∗^*P* < 0.001 compared with the WT group.

**Figure 3:** Increased proliferation and IL-5 production by skin-infiltrating CD4^+^ T cells in female BATF^–/–^ mice. Splenocytes and tail skin-infiltrating mononuclear cells were isolated from 28-week-old female BATF^–/–^ (BATF^–/–^ F) and WT (WT F) mice, followed by flow cytometric analysis. (a) Representative plots and the bar graphs show the percentages of CD4^+^ and CD8^+^cells among CD3^+^TCR*β*^+^ living cells in the spleens and tail skins of female BATF^–/–^ and WT mice. (b–d) Representative plots and the bar graphs show the percentages of Foxp3^+^ (b), Ki67^+^ (c), and IL-5^+^(d) cells within the CD4^+^ living cell populations in the spleens and tail skins of female BATF^–/–^ and WT mice. Data are shown as mean ± standard deviation (SD) and are representative of three independent experiments. ^∗^*P* < 0.05, ^∗∗^*P* < 0.01, and ^∗∗∗^*P* < 0.001 compared with the WT group.

RETRACTED

**Figure 4:** 17*β*-Estradiol induces dermatitis in male BATF^–/–^ mice. Male WT B6 (WT M) and BATF^–/–^ (BATF^–/–^M) mice were injected intraperitoneally with either 1 mg/kg 17*β*-estradiol or sesame oil every 3 days. Estradiol treatment was started at the age of 4 weeks and ended at the age of 24 weeks. (a) A representative image of the tail skins from 2 estradiol-treated BATF^–/–^ mice, 1 sesame oil-treated BATF^–/–^ mouse, and 1 estradiol-treated WT mouse at 24 weeks of age. (b) Macroscopic scores of dermatitis in estradiol-treated BATF^–/–^ (*n* = 16), sesame oil-treated BATF^–/–^ (*n* = 14), and estradiol-treated WT (*n* = 14) male mice at the indicated ages. Statistical significance was determined by two-way analysis of variance (ANOVA). (c) Representative H&E-stained tail skin sections from 24-week-old male BATF^–/–^ and WT mice, which were treated with 17*β*-estradiol or sesame oil as indicated. Scale bars: 400 *μ*m (100× magnification), 200 *μ*m (200× magnification) and 100 *μ*m (400× magnification). (d) Total serum IgE levels detected by enzyme-linked immunosorbent assay (ELISA) from 28-week-old male BATF^–/–^ and WT mice with the indicated treatment (*n* = 20 per group). (e) Relative mRNA expressions of IL-4, IL-5, IL-1*β*, and IFN-*γ* in the tail skins of 28-week-old male estradiol-treated BATF^–/–^, sesame oil-treated BATF^–/–^, and estradiol-treated WT mice. ^∗^*P* < 0.05, ^∗∗^*P* < 0.01, and ^∗∗∗^*P* < 0.001 compared with the WT group.

**Table 1:** Primer sequences used in quantitative real-time PCR.

Gene	Gene ID	Forward primer (5′→3′)	Reverse primer (5′→3′)
*Filaggrin*	*14246*	ATGTCCGCTCTCCTGGAAAG	TGGATTCTTCAAGACTGCCTGTA
*Loricrin*	*16939*	GCGGATCGTCCCAACAGTATC	GCGGATCGTCCCAACAGTATC
*S100A8*	*20201*	AAATCACCATGCCCTCTACAAG	CCCACTTTTATCACCATCGCAA
*S100A9*	*20202*	ATACTCTAGGAAGGAAGGACACC	TCCATGATGTCATTTATGAGGGC
*IFN-γ*	*15978*	ATGAACGCTACACACTGCATC	CCATCCTTTTGCCAGTTCCTC
*TNF-α*	*21926*	CCCTCACACTCAGATCATCTTCT	GCTACGACGTGGGCTACAG
*IL-4*	*16189*	GGTCTCAACCCCCAGCTAGT	GCCGATGATCTCTCTCAAGTGAT
*IL-5*	*16191*	CTCTGTTGACAAGCAATGAGACG	TCTTCAGTATGTCTAGCCCCTG
*IL-22*	*50929*	ATGAGTTTTTCCCTTATGGGGAC	GCTGGAAGTTGGACACCTCAA
*IL-1β*	*16176*	GCAACTGTTCCTGAACTCAACT	ATCTTTTGGGGTCCGTCAACT
*GAPDH*	*14433*	AGGTCGGTGTGAACGGATTTG	TGTAGACCATGTAGTTGAGGTCA

S100A8: S100 calcium-binding protein A8 (calgranulin A); S100A9: S100 calcium-binding protein A9 (calgranulin B); IFN-*γ*: interferon-*γ*; TNF-*α*: tumor necrosis factor *α*; GAPDH: glyceraldehyde-3-phosphate dehydrogenase.

RETRACTED

## Data Availability

The data used to support the findings of this study are included within the article.
